This article has been retracted.

# HLA-B35 and dsRNA Induce Endothelin-1 via Activation of ATF4 in Human Microvascular Endothelial Cells

**DOI:** 10.1371/journal.pone.0056123

**Published:** 2013-02-18

**Authors:** Stefania Lenna, Izabela Chrobak, G. Alessandra Farina, Fernando Rodriguez-Pascual, Santiago Lamas, Robert Lafyatis, Raffaella Scorza, Maria Trojanowska

**Affiliations:** 1 Arthritis Center, Boston University School of Medicine, Boston, Massachusetts, United States of America; 2 Centro de Biología Molecular “Severo Ochoa” (CSIC/UAM), Madrid, Spain; 3 Referral Center for Systemic Autoimmune Diseases, Fondazione IRCCS Ca' Granda Ospedale Maggiore Policlinico and University of Milan, Milan, Italy; University of Pittsburgh, United States of America

## Abstract

Endothelin 1 (ET-1) is a key regulator of vascular homeostasis. We have recently reported that the presence of Human antigen class I, HLA-B35, contributes to human dermal microvascular endothelial cell (HDMEC) dysfunction by upregulating ET-1 and proinflammatory genes. Likewise, a Toll-like receptor 3 (TLR3) ligand, Poly(I:C), was shown to induce ET-1 expression in HDMECs. The goal of this study was to determine the molecular mechanism of ET-1 induction by these two agonists. Because HLA-B35 expression correlated with induction of Binding Immunoglobulin Protein (BiP/GRP78) and several heat shock proteins, we first focused on ER stress and unfolded protein response (UPR) as possible mediators of this response. ER stress inducer, Thapsigargin (TG), HLA-B35, and Poly(I:C) induced ET-1 expression with similar potency in HDMECs. TG and HLA-B35 activated the PERK/eIF2α/ATF4 branch of the UPR and modestly increased the spliced variant of XBP1, but did not affect the ATF6 pathway. Poly(I:C) also activated eIF2α/ATF4 in a protein kinase R (PKR)-dependent manner. Depletion of ATF4 decreased basal expression levels of ET-1 mRNA and protein, and completely prevented upregulation of ET-1 by all three agonists. Additional experiments have demonstrated that the JNK and NF-κB pathways are also required for ET-1 upregulation by these agonists. Formation of the ATF4/c-JUN complex, but not the ATF4/NF-κB complex was increased in the agonist treated cells. The functional role of c-JUN in responses to HLA-B35 and Poly(I:C) was further confirmed in ET-1 promoter assays. This study identified ATF4 as a novel activator of the ET-1 gene. The ER stress/UPR and TLR3 pathways converge on eIF2α/ATF4 during activation of endothelial cells.

## Introduction

Endothelin-1 (ET-1) is a potent vasoconstrictor and one of the key regulators of vascular homeostasis. ET-1 dysfunction is associated with a number of pathological conditions including hypertension, atherosclerosis, cardiovascular disorders, and cancer [1], [2], [3]. Under physiological conditions, ET-1 is produced in small amounts mainly in endothelial cells (ECs). However in pathophysiological conditions, its production is stimulated in a large number of different cell types, including endothelial cells, vascular smooth muscle cells, cardiac myocytes, and inflammatory cells such as macrophages and leukocytes. In addition to its main role as a vasoconstrictor, ET-1 also contributes to inflammation, as well as fibrosis during various pathophysiological processes.

Extensive studies of ET-1 gene expression have led to characterization of the signaling pathways and transcription factors involved in its regulation [4], [5]. A complex network consisting of the common and tissue specific transcription factors responding in the coordinated fashion to physiological and pathological stimuli have been shown to regulate ET-1 expression in a cell type and context specific manner. One of the main regulatory factors is a FOS/JUN complex that binds to an activator protein 1 (AP-1) response element located at a -108 bp in the ET-1 promoter region. This site mediates upregulation of the ET-1 gene by phorbol esters, Angiotensin II, Thrombin, and High-density lipoprotein (HDL), which stimulate AP-1 in a Protein kinase C (PKC)-dependent manner. On the other hand, Leptin activates AP-1 through the Jun N-terminal kinase (JNK) and extracellular-signal-regulated kinases 1/2 (Erk1/2) pathways. AP-1 in cooperation with GATA-binding factor 2 (GATA2) is also required for the basal transcription of the ET-1 gene in endothelial cells, while other members of the GATA family regulate ET-1 expression in other cell types. Additional important transcription binding sites include hypoxia response element, Hypoxia-inducible factors (HIF-1), transforming growth factor β (TGF-β)/Smad response element, which have been also described to cooperate with AP-1 to induce ET-1 [6], as well as the Nuclear factor κB (NF-κB) binding site that mediates responses to inflammatory cytokines. Other cell type specific response elements have also been characterized [7].

Endoplasmic Reticulum (ER) stress is defined as accumulation of unfolded or misfolded proteins in the ER, triggering an adaptive program called the unfolded protein response (UPR). The UPR alleviates ER stress by suppression of protein synthesis, facilitation of protein folding via induction of ER chaperones, and reinforced degradation of unfolded proteins. Three major transmembrane transducers of ER stress have been identified in the ER. Those are the RNA-dependent protein kinase-like ER kinase (PERK), activating transcription factor 6 (ATF6), and inositol-requiring ER-to-nucleus signal kinase 1α (IRE1α). Activation of PERK leads to phosphorylation of the eukaryotic translation initiation factor 2α (eIF2α), causing general inhibition of protein synthesis. In response to ER stress, ATF6 transits to the Golgi where it is cleaved by the proteases Site-1 protease (S1P) and Site-2 protease (S2P), yielding a free cytoplasmic domain which functions as an active transcription factor. Similarly, activated IRE1α catalyzes removal of a small intron from an X-box-binding protein 1 (XBP1) mRNA. This splicing event produces an active transcription factor XBP1. If the cell fails to deal with the protein-folding defect and restore homeostasis, a pro-apoptotic CCAAT/−enhancer-binding protein homologous protein (CHOP)-mediated pathway is initiated [8].

There is extensive evidence that ER stress/UPR is closely linked to the inflammatory pathways through activation of the two key inflammatory mediators, JNK and NF-κB [8], [9] Recent studies have also revealed that UPR and innate immune pathways share common mediators [10], [11]. It was shown that stimulation of the Toll-like receptor (TLR) 2 or TLR4 leads to selective activation of the IRE1a/XBP1 pathway, contributing to the optimal and sustained production of proinflammatory cytokines in macrophages [12]. However, activation of the IRE1α/XBP1 pathway by these TLR agonists did not lead to expression of the genes typically regulated by these mediators during ER stress, suggesting an alternative utilization of the components of the UPR pathways. The specific mechanisms involved in these atypical responses are still not well understood and require further investigation.

We have recently shown that ectopic expression of HLA-B35, an antigen associated with SSc in Choctow Indians [13] and SSc-PAH in Italian patients [14], [15], led to a significant increase of ET-1 and a decrease of eNOS in cultured endothelial cells (ECs) [16]. In addition to ET-1, we have also observed upregulation of interferon-regulated genes and other inflammatory genes in ECs expressing HLA-B35. Furthermore, expression of HLA-B35, but not a control antigen HLA-B8, potently upregulated several cellular chaperones including BiP, HSP70 and HSP40, suggesting an activation of ER stress/UPR in these cells. However, other UPR genes such as ERO1 (ER oxidoreductin 1), and PDI (protein disulphide isomerase), which are involved in oxidative protein folding, as well as a pro-apoptotic UPR mediator, CHOP were not upregulated, consistent with activation of an adaptive phase of the UPR. Relevant to these findings Farina et al have reported upregulation of ET-1 in response to a synthetic analog of dsRNA, Poly(I:C), in dermal endothelial cells and fibroblasts [17]. Given the recently uncovered cross-talk between the UPR and the innate immune pathways, the goal of this study was to further investigate whether common mediators are involved in ET-1 gene regulation in response to these stimuli. Here we report that induction of ER stress or stimulation with Poly(I:C) activate the eIF2α-ATF4 pathway and promote formation of the ATF4/c-JUN complexes. This protein complex in concert with the NF-κB pathway activates ET-1 gene transcription in endothelial cells.

## Materials and Methods

### Reagents

Thapsigargin (TG) was purchased by Sigma-Aldrich (St. Louis, MO). Poly(I:C) was purchased by InvivoGen (San Diego, CA). Tissue culture reagents, EBM kit by Lonza (Walkersville, MD). The protease inhibitor cocktail set III and phosphatase inhibitor cocktail set II were purchased from Calbiochem (San Diego, CA). Enhanced chemiluminescence reagent and bicinchoninic acid protein assay reagent were obtained from Pierce Chemical Co. (Rockford, IL). TRI Reagent was purchased from the Molecular Research Center Inc. (Cincinnati, OH).

For western blot, antibodies were used as followed: goat ATF4 and rabbit ATF6 (Santa Cruz Biotechnology, Santa Clara, CA) at a 1∶500 dilution; rabbit pPERK and PERK (Santa Cruz Biotechnology, Santa Clara, CA) at a 1∶500 dilution, rabbit p-eIF2α and mouse eIF2α Ab (Santa Cruz Biotechnology, Santa Clara, CA) at 1∶500 dilution; rabbit cJun and rabbit NF-κBp65 Ab (Santa Cruz Biotechnology, Santa Clara, CA) at a 1∶500 dilution; monoclonal β-actin Ab (Sigma-Aldrich) at 1∶5000 dilution and mouse Lamin A/C at 1∶1000 dilution.

### Cell Culture

Human dermal microvascular endothelial cells (HDMECs) were isolated from human foreskins using the protocol of Richard et al [18]. Upon informed consent and in compliance with the Institutional Review Board of Human studies, written approval was obtained from Perinatal Committee (IRB number H-29190) of Boston University Medical School. Briefly, primary cultures of human foreskins were established after the removal of epidermis. Such cultures consist of a mixture of HDMECs, dermal fibroblasts, and some keratinocytes. Subconfluent cultures were treated with tumor necrosis factor-α for 6 h to selectively induce the expression of E-selectin in HDMECs. HDMECs were then purified using magnetic beads coupled to an anti-E-selectin monoclonal antibody. First passage cultures usually consist of >99% HDMECs. A second immunomagnetic purification step ensures homogenous population of HDMECs suitable for long term culturing. Purity of the HDMEC cultures was evaluated using anti-CD31 and anti-von Willebrand factor antibodies. These cells were cultured on collagen-coated 6-well plate in EBM medium supplemented with 10% FBS, EC growth supplement mix at 37°C under 5% CO2 in air. The culture medium was changed every other day. HDMECs harvested between passage 2 and 6 were used for experiments.

### Adenoviral Constructs

An adenoviral vector expressing HLA-B35 (or Ad-B8) and control green fluorescent protein (Ad-Go) were generated as described earlier [18]. The dose used to transduce human dermal microvascular endothelial cells was 10 multiplicities of infection of the adenovirus (MOI). ECs grown in a 6-well dish were transduced with Ad (Ad-B35/GFP, -B8/GFP, and -GFP), after 48 h cells were collected for RNA analyses or for Western blot.

### Real-time PCR

Total RNA was extracted using the guanidiniumthiocyanate-phenol-chloroform method, concentration and purity was determined by measuring OD at 260 and 280 nm using a spectrophotometer. RNA was reversibly transcribed by aid of the first-strand cDNA Synthesis Kit for RT-PCR (Roche Applied Science, Indianapolis, IN). To avoid amplification from traces of possible DNA contamination in the RNA isolation, PCR primers were designed to span introns. All primers were checked for specificity by Blast search. Real-time RT-PCR was performed using IQ SYBR Green Supermix (Bio-Rad, Hercules, CA) and MyiQ Single-Color Real-Time PCR Detection System (Bio-Rad). The amount of template used in the PCR reactions was cDNA corresponding to 200 ng reverse-transcribed total RNA. DNA polymerase was first activated at 95°C for 3 min, denatured at 95°C for 30 s, and annealed/extended at 61°C for 30 s, for 40 cycles according to the manufacturer's protocol. Expression of the housekeeping gene β-actin served as an internal positive control in each assay performed. After measurement of the relative fluorescence intensity for each sample, the amount of each mRNA transcript was expressed as a threshold cycle value. The primers are listed in **Table 1**.

**Table 1:** Primer sequences for quantitative PCR.

	Forward	Reverse
**Human-PPET-1**	5′-gctcgtccctgatggataaa-3′	5′-ccatacggaacaacgtgct-3′
**Human-ATF4**	5′-tggctggctgtggatgg-3′	5′-tcccggagaaggcatcct-3′
**Human-ATF6**	5′-ttttagcccgggactctttc-3′	5′-tcagcaaagagagcagaatcc-3′
**Human-XBP1u**	5′-ccttgtagttgagaaccagg-3′	5′-gggcttggtatatatgtgg-3′
**Human-XBP1s**	5′-ggtctgctgagtccgcagcagg-3′	5′-gggcttggtatatatgtgg-3′
**Human-PKR**	5′-tgttgggatggatttgattatg-3′	5′-gaaaaggcacttagtctttgacct-3′
**Human-βactin**	5′-aatgtcgcggaggacctttgattgc-3′	5′-aggatggcaagggacttcctgtaa-3′
**Mouse-ATF4**	5′-gagcttcctgaacagcgaagtg-3′	5′-tggccacctccagatagtcatc-3′
**Mouse-βactin**	5′-ctaaggccaaccgtgaaaag-3′	5′-accagaggcatacagggaca-3′

### Immunofluorescence Staining on Adherent Cell Cultures

Cultured HDMECs grown on collagen-coated cover slips were transduced with Adenovirus carrying HLA-B35 (Ad-B35/GFP), Ad-B8/GFP and Ad-G0/GFP (virus control) for 48 hours. Treated cells were fixed with 4% paraformaldehyde for 15 minutes followed by incubation with 0.15 M Glycine for 30 min. Non-specific protein binding was blocked with 3% BSA for 1 h. Next, cells were incubated at 4°C overnight with primary mouse monoclonal MHC class I Ab (W6/32) (Santa Cruz Biotechnology, Santa Clara, CA) at a 1∶500 dilution. After washing, cell cultures were incubated with Alexa fluor 594 donkey anti-mouse (Invitrogen, Grand Island, NY) antibody for 1.5 h. Cells were mounted on slides using Vectashield with DAPI (Vector Laboratories, Burlingame, CA) and examined using a FluoView FV10i confocal microscope system (Olympus, Center Valley, PA) at 488 nm (green), 594 nm (red) and 405 nm (blue).

### Western Blot Analysis

Cells were collected and washed with PBS. Cell pellets were suspended in lysis buffer containing 20 mM Tris-HCl, pH 7.5, 15 mM NaCl,1 mM EDTA, 1 mM EGTA, 1% Triton X-100, 2.5 mM sodium pyrophosphate, and 1 mM glycerophosphate with freshly added phosphatase inhibitors (5 mM sodium fluoride and 1 mM Na3VO4) and a protease inhibitor mixture (Sigma-Aldrich). Protein concentration was quantified using the BCA Protein Assay kit (Pierce). Equal amounts of total proteins per sample were separated via SDS-PAGE and transferred to nitrocellulose membranes (Bio-Rad). Membranes were blocked in milk in TBST overnight at 4°C and probed with primary Ab overnight at 4°C. After TBST washes, membranes were probed with HRP-conjugated secondary Ab against the appropriate species for 1–2 h at room temperature. Protein levels were visualized using ECL reagents (Amersham Biosciences, Piscataway, NJ).

### ET-1 Bio-assay

The ET-1 bioassay was performed according to the protocol supplied with the kit from Assay Designs (cat no. 900-020A). Standards and samples were incubated in supplied pre-coated 96-well plate, washed, incubated with horse radish peroxidase labeled anti- ET-1 antibody and washed again before adding the provided TMB substrate and measuring the absorbance.

### siRNA Experiments

HDMECs were trasfected with either siRNA specific to human ATF4 (ON-TARGET plus SMARTpool, Dharmacon RNA Technologies, CO), PKR (Santa Cruz biotechnology, CA) or negative-control siRNA (Qiagen, Chatsworth, CA) at concentration of 20 nM using HiPerfect reagent (Qiagen) according to the manufacturer's protocol. After 48 hours, RNA was extracted and Real-time PCR was performed.

### Inhibitor Experiment

HDMECs were incubated in the presence of the 25 nM of JNK SP600125 or NF-κB SN50 inhibitor (Enzo Life Sciences, Farmingdale, NY) for 3 hours before treatment. After 48 hours, RNA and protein were extracted.

### Co-Immunoprecipitation

Cell lysates were prepared after appropriate treatment in radioimmune precipitation buffer. For immunoprecipitation of cJUN (or NF-κB p65), antibody was added to 300 µg of precleared cell lysate, and complex formation was carried out at 4°C overnight. The protein-antibody complexes were recovered using protein G-Sepharose beads for 2 h at 4°C. The immunoprecipitates were washed four times in radioimmune precipitation buffer, eluted by boiling for 5 min in 2× SDS sample buffer, and analyzed by Western blot with anti-ATF4 antibody (Santa Cruz Biotechnology, Inc., Santa Cruz, CA).

### Plasmids, Transient Transfections and Luciferase Assay

Luciferase reporters driven by −650-bp and −193-bp fragments (representing the wildtype and mutated AP-1 site) of the human ET-1 promoter described previously 1. Transient transfections of promoters were performed in HDMECs seeded into 6-well plates using Fugene6 (Roche Applied Science) according to the manufacturer's instructions. After overnight incubation, cells were treated and then further incubated for 24 h. The cells were harvested and assayed for luciferase reporter activity using the Promega luciferase assay kit according to the manufacturer's instructions. Promoter/reporter plasmids were cotransfected with pCMV-βGal (Clontech), which was used to adjust for differences in transfection efficiencies between samples. Cells were harvested and Luciferase activity of the promoter was assayed using Promega Luciferase assay kit. Values given are means ± standard errors of triplicate assays from three individual experiments.

### In vivo Administration of Poly(I:C)

C57Bl/6 WT and C57Bl/6 TICAM/TRIF −/− mice were obtained from The Jackson Laboratory; C57Bl/6 IFNAR1−/− mice were provided by Dr John Sprent. All of the experiments were performed under the guidelines of the Boston University Institutional Animal Care and Use Committee. Osmotic pumps designed to deliver Poly(I:C) (0.5 mg/ml in PBS, 0.1 mg total dose in 200 µl released over 7 days, Alzet) or PBS were implanted subcutaneously on the back in 6–10-weekold mice. After 7 days mice were killed and skin (∼1 cm2) surrounding the pump outlet was homogenised in Trizol for preparation of RNA, then minced and disrupted using a Polytron homogeniser and processed according to the manufacturer's protocol.

This study was carried out in strict accordance with the recommendations in the Guide for the Care and Use of Laboratory Animals of the National Institutes of Health. The protocol was approved by the Committee on the Ethics of Animal Experiments of the Boston University (Permit Number: AN-14942.2012.01). All surgery was performed under sodium pentobarbital anesthesia, and all efforts were made to minimize suffering.”.

### Immunostaining

Skin sections biopsies from healthy individuals and limited cutaneous systemic sclerosis (lcSSc) patients including 8 patients with pulmonary arterial hypertension (lcSSc-PAH) based on echoradiography and right heart catheterization and 11 patients without PAH (lcSSc-noPAH) and 5 healthy controls were provided by the Boston University Core Centers (http://www.bu.edu/sscores/); IRB: H31–506. Patient information is included in Table 2. Immunohistochemistry was performed on formalin-fixed, paraffin-embedded tissue sections using a Vectastain ABC kit (Vector Laboratories, Burlingame, CA) according to the manufacturer’s instructions. Briefly, 8-micrometer-thick sections were mounted on APES (amino-propyl-triethoxy-silane)-coated slides, deparaffinized with Histo-Clear (National diagnostic, Atlanta GA), and rehydrated through a graded series of ethanol. Endogenous peroxidase was blocked by incubation in 0.3% hydrogen peroxide for 15 minutes and incubated with blocking buffer for 1 hour. The sections were then incubated overnight at 4°C with antibody against ATF4 (Abcam, Cambridge, MA) diluted 1∶500 in blocking serum, followed by the incubation with secondary antibody. The concentration of primary antibody was first tested to determine the optimal sensitivity range. The immunoreactivity was visualized with diaminobenzidine (Vector laboratories, Burlingame, CA) and the sections were counterstained with hematoxylin.

**Table 2:** Clinical and hemodynamic data of study subjects.

	Sample	Age	Gender	DiseaseDuration	PAP	PCWP	PASP	Treatment	ATF4 staining
Normal	11-6	30	M						++
Normal	11-7	24	M						+
Normal	11-8	47	F						++
Normal	12-1	25	M						−
Normal	12-2	25	F						+
lcSSc PAH	12-8	65	F	16 years 1 month	49	30	44	no medications	−
lcSSc PAH	12-7	58	M	16 years	30	12	65	no medications	++
lcSSc PAH	12-6	69	F	16 years	54	5	71	no medications	++
lcSSc PAH	12-3	75	F	25 years	48	9–10	62	sildenafil	+
lcSSc PAH	12–17	30	F	1 years 8 months	25	2	N/A	cell cept revatio	+
lcSSc PAH	12–20	60	F	3 years	25	2	N/A	prednisone	+++
lcSSc PAH	12–18	59	F	15 years	N/A	N/A	N/A	none	+
lcSSc PAH	12–19	52	F	25 years	N/A	N/A	N/A	viagra	++
lcSSc NoPAH	12–27	59	M				45	none	**+**
lcSSc NoPAH	12-2	65	F	10 years				myocophenolate	+
lcSSc NoPAH	12-10	40	F	2 years				none	**++**
lcSSc NoPAH	12-1	58	F	2 years				prednisone, mycophenolate	−
lcSSc NoPAH	12–35	56	F	8 years			33	none	+
lcSSc NoPAH	12–31	61	F	14 years				hydroxychloroquine	+
lcSSc NoPAH	12–28	65	F	6 months			25	none	−
lcSSc NoPAH	12–25	67	M	7 years			25	none	+
lcSSc NoPAH	12–10	40	F	2 years				cyclophosphamide	++
lcSSc NoPAH	12–13	39	F	1 year				cytoxan	+
lcSSc NoPAH	12–21	20	F	6 years				none	++

PAP = pulmonary artery pressure. PCWP = pulmonary capillary wedge pressure. PASP = pulmonary artery systolic pressure.

− indicates no staining or little staining in <10% of the cells.

+ indicates faint, partial staining in >20% of the cells.

++ indicates light to moderate stain in >50% of the cells.

+++ indicates bright staining in >50% of the cells.

### Statistical Analysis

Student's t test analysis was performed to determine statistical significance. Values less than or equal to 0.05 were considered statistically significant. All experiments were repeated at least three times using independently isolated endothelial cell cultures.

## Results

### ER Stress and Poly(I:C) Activate Common ER Stress/UPR Pathways in HDMECs

In the initial experiment we compared the effects of HLA-B35 with a known ER stress inducer, thapsigargin (TG), and a TLR3 agonist, Poly(I:C), on the expression of ET-1 mRNA and protein in primary dermal microvascular endothelial cells (HDMECs). HLA-B35 was expressed using adenoviral delivery as previously described [16]. To control for the presence of adenoviral genes we used adenovirus expressing a closely related antigen, HLA-B8, as well as an empty virus. As shown in Fig. 1a, HLA-B35 and Poly(I:C) upregulated (pre-pro-endothelin-1) PPET-1 mRNA levels with a similar potency 7-fold ±0.58, p  = 0.05 vs 8-fold±0.25, p = 0.05, respectively, while TG was a stronger inducer of PPET-1 (26-fold ±0.75, *p*  = 0.001). Ad-HLA-B8, as well as an empty virus vector (data not shown) did not affect PPET1 mRNA expression. To verify that the increase in PPET-1 mRNA corresponds to an increase of the bioactive 21-aa ET-1 peptide, we measured levels of ET-1 protein in supernatants of Ad-B35 (and Ad-B8), TG and TLR ligand-treated ECs. Consistent with the mRNA measurements ER stress inducers increased ET-1 protein levels (Ad-B35, 3.5-fold±0.6, p = 0.05 and TG, 5.3-fold±0.80, p = 0.05). Similarly, Poly(I:C) induced ET-1 protein by 3.7-fold±0.98 (Fig. 1b). PPET-1 mRNA expression was further enhanced by a combination of HLA-B35, and to a lesser degree TG, and Poly(I:C) (Fig. 1c).

**Figure 1:** HLA-B35, TG, and Poly(I:C) upregulate ET-1 mRNA and protein in HDMECs. Upregulation of PPET-1 mRNA after HLA-B35 (or HLA-B8), TG, or Poly(I:C) treatments alone (a) or in combination (c) in HDMECs. Confluent dishes of HDMECs were transduced with 10 MOI of Adenovirus encoding HLA-B35/GFP (Ad-HLA-B8/GFP) for 48 h or treated with 10pM TG, or 2.5 µg/µl Poly(I:C) for 24 hours. Total RNA was extracted and mRNA levels of PPET-1 were quantified by quantitative RT-PCR. Expression of the housekeeping gene β-actin served as an internal positive control in each assay performed. After measurement of the relative fluorescence intensity for each sample, the amount of each mRNA transcript was expressed as a threshold cycle value. (b) Bioactive 21-aa ET-1 peptide in HDMECs after Ad-B35/GFP (Ad-B8/GFP), TG, or Poly(I:C) treatment. ET-1 protein was measured by ELISA in the supernatants. The average protein concentration for each group is represented as a bar ± SE. *p  = 0.05; **p  = 0.001 **(d)** Immunofluorescence was performed using mouse monoclonal MHC class I Ab (W6/32) in HDMECs transduced with HLA-B35 (Ad-B35/GFP), Ad-B8/GFP and Ad- G0/GFP (virus control). Left column DAPI, middle column GFP, right column HLA. Bar: 100 µm.

To further determine if HLA-B35 mediates its effects via peptide binding to the antigen-binding groove we utilized mouse monoclonal anti-MHC class I blocking antibody (W6/32). HDMECs transduced with Ad-HLA-B35/GFP and HLA-B8/GFP for 24 hours were treated with increasing dose of W6/32 (0.1–10 µg/ml) for the following 24 hours. Treatment with antibody did not affect ET-1 mRNA levels, suggesting that HLA-B35 does not modulate ET-1 through peptide binding to the antigen-binding groove (supplemental data, Fig. S1). To determine subcellular localization of ectopic HLA-B35 we performed immunofluorescence staining using HDMECs transduced with Ad-HLA-B35/GFP, Ad-HLAB8/GFP and Ad-G0/GFP (virus control) for 48 hours. Spotty positive staining was observed in the cytoplasm primarily around the nucleus, suggesting ER retention of the HLA-B35 and HLA-B8. Together, these data suggest that HLA-B35 is primarily retained in the ER, where it might induce ER stress and UPR. Interestingly, although HLA-B8 displayed a similar cellular distribution, expression of HLA-B8 was not associated with upregulation of BiP and other heat shock proteins [18]. The specific structural determinants of HLA-B35 that may explain its biological effects are currently not known.

To further characterize the nature of the HLA-B35-mediated ER stress, we examined the effect of HLA-B35 (or HLA-B8), TG, and Poly(I:C) on the mRNA expression of the three main UPR mediators, transcription factors ATF4, ATF6 and XBP1. ATF4 mRNA levels were significantly increased in response to the HLA-B35 and Poly(I:C) treatment, while TG was a less potent inducer of ATF4 mRNA under this experimental conditions (Fig. 2a). When Poly(I:C) was used in combination with the ER stress inducers, a further upregulation of ATF4 mRNA was observed (Fig. 2b). Furthermore, both HLA-B35 and TG moderately increased spliced (active) form of the transcription factor XBP1 (XBP1s), while TLR3 had no effect on the XBP1 splicing (Fig. 2c). In contrast, the expression level of ATF6 was not responsive to any of these treatments in HDMECs (Fig. 2d).

**Figure 2:** ER stress and Poly(I:C) activate selected ER stress/UPR pathways. ATF4 (a, b), XBP1 splicing (c) and ATF6 (d) mRNA levels in HDMECs treated with HLA B35 (HLA-B8), TG, and Poly(I:C) alone or in combination. Confluent dishes of HDMECs were transduced with 10 MOI of Ad-B35/GFP (or Ad- B8/GFP) for 48 h treated with 10pM TG, or 2.5 µg/µl Poly(I:C) for 24 hours. Total RNA was extracted and mRNA levels of transcription factors were examined by quantitative RT-PCR. Expression of the housekeeping gene β-actin served as an internal positive control in each assay performed. After measurement of the relative fluorescence intensity for each sample, the amount of each mRNA transcript was expressed as a threshold cycle value. *p  = 0.05; **p  = 0.001.

Since nuclear translocation of ATF4 is indicative of its activation status, we examined nuclear extracts for the presence of ATF4 by western blot. Nuclear ATF4 was examined at various time points (15 min. to 6 hours) after TG and Poly(I:C) treatments and 24 hours post infection with HLA-B35 or HLA-B8 adenoviruses. Nuclear ATF4 was rapidly increased (15–30 min) after TG and Poly(I:C) treatments (Fig. 3a and Fig. 3b). Likewise, HLA-B35 markedly increased nuclear presence of ATF4 (Fig. 3c). Furthermore, increased phosphorylation of the upstream activators of ATF4, PERK and eIF2α, was observed in response to these treatments (Fig. 3, right panels). Consistent with the mRNA data, nuclear levels of ATF6 remained unchanged. Together, these results demonstrate that ATF4 is activated in a similar manner by ER stress/UPR and Poly(I:C) in endothelial cells.

**Figure 3:** ER stress and Poly(I:C) activate ATF4 nuclear translocation and enhance phosphorylation of PERK and eIF2α. ATF4**,** pPERK/PERK, and p-eIF2α**/**eIF2α protein levels in HDMECs after treatment with 10pM TG (a), 2.5 µg/µl Poly(I:C) (b), or transduction with 10 MOI of HLA-B35 or HLA-B8 Ads for 48 hours (c). 20 µg of nuclear extract were separated via 15% SDS-PAGE for ATF4 and 10% SDS-PAGE for ATF6. 20 µg of total cellular proteins were separated via 15% SDS-PAGE for pPERK/PERK and 10% SDS-PAGE for peIF2α/eIF2α, then transferred to a nitrocellulose membrane. The blots were probed overnight with primary Abs at 4°C. As a control for equal protein loading, membranes were stripped and reprobed for Lamin A/C or β-actin. Representative blots from at least three independent experiments are shown.

### PKR Mediates Activation of the ET-1 Gene in Response to Poly(I:C)

Protein kinase RNA-activated (PKR) is activated by dsRNA and plays an important role in the IFN signaling [19]. Similar to PERK, activated PKR induces phosphorylation of eIF2α and a subsequent ATF4 nuclear translocation. To clarify whether activation of PKR is involved in the ET-1 upregulation by Poly(I:C) treatment, we used siRNA approach to knock down PKR. Initial experiments have established an optimal dose and time for PKR siRNA to achieve maximal inhibition of the PKR mRNA level. Treatment of HDMECs with 20 nM of PKR siRNA for 48 hours resulted in depletion of PKR mRNA levels (around 50%) (Fig. 4a). Following 24 hour incubation with siRNA, cells were treated with Poly(I:C) for additional 24 hours. Under these conditions basal PPET-1 gene expression was downregulated by the siRNA treatment, suggesting that PKR contributes, in part, to the constitutive expression of ET-1 (Fig. 4b). Furthermore, depletion of PKR almost completely abrogated Poly(I:C)-induced stimulation of PPET-1 (Fig. 4b). Interestingly, depletion of PKR upregulated phosphorylated eIF2α (Fig. 4c), as well as nuclear ATF4 level (Fig. 4d) in unstimulated cells, suggesting that without activation, PKR may negatively regulate this pathway. However, in the Poly(I:C)-stimulated cells phosphorylation of eIF2α was abrogated and the ATF4 nuclear level was markedly decreased. These results suggest that PKR mediates ET-1 upregulation in response to Poly(I:C) in HDMECs.

**Figure 4:** Poly(I:C) induces ET-1 gene through the PKR-dependent activation of the eIF2α/ATF4 pathway. 80% confluency, HDMECs were treated with 20 nM PKR siRNA (siSCR) with or without Poly(I:C) treatment (a and b). Total RNA was extracted and mRNA level of PKR (a) and PPET1 (b) were quantified by quantitative RT-PCR. Expression of the housekeeping gene β-actin served as an internal positive control in each assay performed. After measurement of the relative fluorescence intensity for each sample, the amount of each mRNA transcript was expressed as a threshold cycle value. 20 µg of nuclear extract were separated via 15% SDS-PAGE for ATF4 (c), 20 µg of total cell lysate were separated via 10% SDS-PAGE for peIF2α/eIF2α (d), then transferred to a nitrocellulose membrane. The blots were probed overnight with primary Abs at 4°C. As a control for equal protein loading, membranes were stripped and reprobed for Lamin A/C or β-actin. Representative blots of at least three experiments are shown. (e) Expression of ATF4 by real-time PCR analysis of skin mRNA from C57B1/6 WT (n = 10), C57B1/6 IFNAR1−/− (n = 8) and C57B1/6 TRIF/TICAM −/− (n = 6) mice 1 week after subcutaneous insertion of osmotic pumps containing Poly(I:C). Fold-change shown in the graphs is normalized to mRNA expression by one of the control mice. *p  = 0.05; **p  = 0.001 (f) ATF4 protein expression in dermal biopsies obtained from C57Bl/6 WT mice 1 week after subcutaneous insertion of osmotic pumps containing Poly(I:C) or PBS (as control), and processed for immunohistochemistry as described under Methods. Representative images of microvessels from PBS and Poly(I:C) skin is shown. Bar: 20 µm, 10 µm.

We next investigated whether ATF4 is involved in regulation of ET-1 in the Poly(I:C)-treated mice. It has been previously reported that mice receiving continuous Poly(I:C) injection through the osmotic pump for 7 days showed highly increased expression of ET-1 [17]. In addition, this response was abrogated in the TIR-domain-containing adapter-inducing interferon β/Toll-interleukin 1 receptor domain (TIR)-containing adaptor molecule-1 (TRIF/TICAM) deficient mice, and only partially inhibited in the interferon-α/β receptor (IFNAR)-1 deficient mice, indicating that ET-1 induction following Poly(I:C) stimulation is mediated by TLR3. As shown in Fig. 4e, expression of ATF4 closely correlated with the previously shown ET-1 expression in the Poly(I:C) treated mice [16]. Increased expression of ATF4 mRNA was also observed in the Poly(I:C) treated WT mice, but this response was significantly decreased in the TRIF/TICAM−/− mice [WT Poly(I:C) vs TRIF/TICAM−/− Poly(I:C) p = 0.001]. On the other hand, depletion of IFNAR1 had only a modest, non-significant inhibitory effect on the Poly(I:C)-induced ATF4 mRNA level in comparison to WT mice. We next examined the distribution of ATF4 protein in the mouse skin by immunohistochemistry. Analyses of skin showed ATF4 staining in vascular endothelial cells in mouse skin after 1 week of Poly(I:C) infusion, and no staining in PBS infused skin. Unfortunately there were only few visible vessels in the sections analyzed (Fig. 4f).

### ATF4 is Required for the Upregulation of ET-1 in Response to HLA-B35/ER Stress and Poly(I:C) in HDMECs

In order to determine whether ATF4 is directly involved in the regulation of ET-1 gene we employed a siRNA approach to knock down ATF4. Initial experiments established an optimal dose and time for the ATF4 siRNA to achieve maximal inhibition of endogenous ATF4 mRNA level. Treatment of HDMECs with 20 nM ATF4 siRNA for 48 hours resulted in depletion of ATF4 mRNA levels (up to 50–60%) (Fig. 5a). Under these conditions basal expression levels of ET-1 mRNA and protein were also consistently decreased by ∼30% (Fig. 5c and d). Following 24 hour incubation with siRNA, cells were treated with Ad-B35/GFP (or Ad-B8), TG and Poly(I:C) for additional 24 hours. Depletion of ATF4 completely abolished upregulation of ET-1 mRNA (Fig. 5b) and protein (Fig. 5c) in response to these treatments, suggesting that ATF4 is required for these responses.

**Figure 5:** ER stress and Poly(I:C) upregulate ET1 via ATF4. 80% confluency, HDMECs were treated with 20 nM ATF4 siRNA (or siSCR) prior to treatment with HLA-B35 (HLA-B8), TG, or Poly(I:C). Total RNA was extracted and mRNA level of ATF4 (a) and PPET-1 (b) were quantified by quantitative RT-PCR. Expression of the housekeeping gene β-actin served as an internal positive control in each assay performed. After measurement of the relative fluorescence intensity for each sample, the amount of each mRNA transcript was expressed as a threshold cycle value. (c) ET-1 protein was measured by ELISA in the supernatants (n = 2). The average ET-1 protein concentration for each group is represented as a bar ± SE. *p  = 0.05; **p  = 0.001. (d) ATF4 protein expression in human skin microvessels. Lesional skin biopsies were obtained from patients with lcSSc (with and without PAH) and healthy controls, and processed for immunohistochemistry as described under Methods. Representative images of microvessels from healthy control and lcSSc patients are shown; similar immunostaining pattern was observed in control and lcSSc skin biopsies. Bar: 50 µm, 10 µm.

We next examined the distribution of ATF4 protein in the human skin by immunohistochemistry. Analyses of skin microvessels showed heteregoneus distribution of ATF4, with some vessels exhibiting strong endothelial cell nuclear staining, while other vessels were negative for ATF4 (Fig. 5d). The number of positive vessels also varied between different individuals. Because patients with SSc have elevated circulating levels of ET-1 [20] we also analyzed skin samples obtained from 19 patients with limited cutaneous SSc (lcSSc), including 8 patients with PAH (lcSSc-PAH), and 11 lcSSc-noPAH. Similar to healthy control skin, endothelial cell expression of ATF4 varied between the patients, however there was no overall difference in the intensity or staining pattern between lcSSc and healthy individual biopsies. We did not have information regarding the level of circulating ET-1 or the presence of HLA-B35 antigen in this group of patients. Together, these data indicate that ATF4 is highly expressed in a subset of dermal microvessels, where it is likely involved in responses to various environmental stimuli.

### JNK and NF-κB Contribute to the ER Stress and Poly(I:C) Induction of ET-1

JNK and NF-κB pathways have been previously reported to contribute to the ET-1 gene expression in response to various stimuli [4], [5]. To determine if JNK and NF-κB contribute to the upregulation of ET-1 in response to ER stress and TLR3 agonists, cells were treated with HLA-B35, TG, and Poly(I:C) in the presence or absence of the pharmacological inhibitors of these pathways. Treatment with JNK inhibitor (SP6001, 25 nM) resulted in down regulation of the basal and agonist-induced PPET-1 mRNA levels (Fig. 6a, top panel). On the other hand**,** basal expression of PPET-1 mRNA was not affected by the NF-κB inhibitor (SN50, 25 nM), however stimulation of PPET1 by HLA-B35, TG, and Poly(I:C) was completely inhibited (Fig. 6b, top panel http://www.nature.com/jid/journal/v128/n8/full/jid200839a.html - fig. 1). Similar results were observed at the protein levels (Fig. 6a and b, bottom panels). Interestingly, while stimulation of ET-1 by HLA-B35 or TG was similarly affected by the inhibitors of the JNK and NF-κB pathways, Poly(I:C) stimulation of ET-1 was particularly sensitive to depletion of the NF-κB pathway, suggesting that NF-κB plays a predominant role in activation of the ET-1 gene by Poly(I:C) in HDMECs.

**Figure 6:** JNK and NF-κB contribute to the ER stress and Poly(I:C) induction of ET-1. Cells were treated with 25 nM of JNK (a) or NF-κB (b) inhibitors for 3 hours before HLA-B35 (HLA-B8), TG, or Poly(I:C) treatments. Total RNA was extracted and mRNA levels of PPET-1 were quantified by quantitative RT-PCR (top panel). ET-1 protein was measured by ELISA in the supernatants (bottom panel). The average protein concentration for each group (n = 2) is represented as a bar ± SE *p  = 0.05; **p  = 0.001.

### ATF4/c-JUN Complexes Mediate ET-1 Induction by ER Stress and Poly(I:C)

ET-1 gene promoter contains binding sites for a number of transcription factors, however using bioinformatics tools we were unable to locate consensus ATF4 binding site within the promoter region. Based on the previous report identifying ATF4 as a partner of c-JUN in a two-hybrid screen [21], we asked whether ATF4 could form protein complexes with c-JUN in HDMECs. As shown in Fig. 7a, ATF4/c-JUN complexes were present in unstimulated cells and were increased upon stimulation with HLA-B35, TG, and Poly(I:C). While, we could also detect formation of the ATF/NF-κB complexes in unstimulated cells, formation of these complexes was not affected by the agonists (Fig. 7b), suggesting that formation of the ATF4/c-JUN complexes is not simply driven by the elevated levels of ATF4 in stimulated cells.

**Figure 7:** Transcriptional upregulation of ET-1 by ER stress and Poly(I:C) is mediated through the ATF4/cJUN complex. Cell lysates from the HLA-B35 (HLA-B8), TG, or Poly(I:C) treated HDMECs were immunoprecipitated with cJUN (a) or NF-κB p65 antibodies (b) and then analyzed for ATF4 by western blot. Cells were transfected with the luciferase reporter driven by the −650/+172–bp fragment of the human ET-1 promoter (c) or with the −193-bp ppET-1-prom-luc construct (wild type) or constructs with specific mutations in the AP-1 binding site (d). 24 hours post transfection with the indicated plasmids, cells were stimulated with HLA-B35 (HLA-B8) Ads, TG and Poly(I:C) for an additional 24 h. Transfections were normalized using pSVgalactosidase control vector. Basal and induced luciferase activity was measured by luminometry. The graph represents fold change in promoter activity in response to various treatments in comparison with control promoter, which was arbitrarily set at 1. (e) Schematic diagram showing PKR and PERK induced activation of the eIF2α-ATF4 axis followed by the protein complex formation with c-JUN and induction of the ET-1 gene transcription through the AP1 response element.

We next utilized human ET-1 promoter constructs consisting of the −650/+172–bp fragment fused to the luciferase reporter gene to confirm functional role of ATF4 in regulation of the ET-1 gene. Transcriptional activation of the ET-1 promoter was observed after treatment with HLA-B35, TG, and Poly(I:C) (Fig. 7c). To analyze whether AP1 binding site was required for the regulation of ET-1 transcription, cells were transfected with the 193-bp ET-1-prom-luc construct (wild type) or the same construct carrying mutated AP-1 binding site. As shown in Fig. 7d, mutation in the AP1 binding site reduced the ER stress and Poly(I:C) induction of the ET-1 promoter. These results support the functional role of the AP1 complex in the ER stress and Poly(I:C)-mediated induction of the ET-1 gene expression.

## Discussion

In this study we show for the first time that ATF4 is a novel regulator of the ET-1 gene in endothelial cells. ATF4 contributes to the basal expression of ET-1 and is required for the induction of ET-1 in response to both ER stress and dsRNA. Our results strongly suggest that activation of the eIF2α/ATF4 pathway leads to increased formation of the ATF4 protein complexes with c-JUN, which, in turn, activate ET-1 transcription through the AP1 response element. ER stress inducers, including HLA-B35 and TG, as well as dsRNA, also upregulate mRNA and protein expression of ATF4, thus further amplifying this signaling pathway (see diagram, Fig. 7e). Additional experiments show that NF-κB, which is also activated by the ER stress and dsRNA in HDMECs, contributes to the activation of ET-1 gene expression. Interestingly, although, ATF4 forms protein complexes with NF-κB in HDMECs, formation of these complexes was not increased by the stimuli used in our study. Since NF-κB plays a key role in activation of the ET-1 gene by cytokines, it is possible that the ATF4/NF-κB complexes are involved in those responses. Together, this study identifies ATF4 as a key mediator of ET-1 gene activation in response to cellular stress.

ATF4 is a short-live, basic region-leucine zipper (bZip) protein that belongs to a family of the ATF/CREB transcription factors [22]. Under normal physiological conditions translation of the ATF4 protein is inefficient due to the presence of a short open reading frame in its 5′ untranslated region; however ATF4 protein translation is facilitated by various stress conditions that trigger global inhibition of protein synthesis [22]. Such conditions, including ER stress, viral infection, nutrient starvation, and low levels of heme induce activation of distinct protein kinases that in turn lead to phosphorylation of a common downstream mediator, eIF2αβresulting in translational repression. The known kinases that phosphorylate eIF2α include ER stress induced PERK, dsRNA induced PKR, as well as GCN2 (general control non repressed 2) and heme regulated inhibitor, HRI [22]. Here we show that stimulation of ET-1 in response to Poly(I:C) is mediated by PKR. In a related study Gargalovic et al have reported activation of the eIF2α-ATF4 in human atherosclerotic lesions and in cultured aortic endothelial cells exposed to oxidized phospholipids [10]. The authors demonstrated that ATF4 contributed to the upregulation of several inflammatory cytokines in cultured aortic endothelial cells. ATF4 was also upregulated by herpesvirus 8 infection and contributed to proangiogenic response via MCP1 upregulation [23]. Furthermore, rapid induction of ATF4 has been observed in smooth muscle cells (SMCs) in the medial compartment of balloon injured rat carotid arteries [24]. Additional studies with cultured SMCs have demonstrated that Fibroblast growth factors (FGF)-2 and mechanical injury stimulate ATF4 levels, and that ATF4 is required for the FGF-2 mediated upregulation of Vascular endothelial growth factor (VEGF)-A [24]. Our study indicates that ET-1 is among the target genes positively regulated by the eIF2α-ATF4 axis in response to ER stress in endothelial cells. Collectively, these studies support a key role for the eIF2α-ATF4 pathway in response to vascular injury [25].

TLR3 is recognized by viral double-stranded RNA (dsRNA) or its synthetic analog, Poly(I:C), and is expressed on the cell membrane or in the intracellular vesicles, depending on the cell type [26], [27]. Ligand binding to the dimerized TLR3, leads to recruitment of an adaptor protein TRIF/TICAM, which functions as a platform for binding of additional signaling molecules and activation of type I interferon and NF-κB pathways [27]. Previous studies have shown that activation of TLR3 signaling is harmful to endothelial cells by promoting inflammatory and atherogenic response *in vitro* and causing impairment of vessel regeneration in vivo [28]. Elevated levels of TLR3 were found on fibroblasts, immune and endothelial cells in SSc skin biopsies, thus implicating this pathway in the pathogenesis of SSc [29], [30]. This study extends previous work from our group that demonstrated activation of the markers of vascular injury by dsRNA/Poly(I:C) and potential role of the TLR3 signaling to the pathogenesis of SSc [16]. Several studies have shown that activation of the TLR3 signaling pathway leads to impairment of the endothelial cell function including activation of proinflammatory and pro-atherosclerotic mechanisms [31], [32]. ER stress/UPR, as well as the activation of the innate immunity pathways has been implicated in the pathogenesis of several inflammatory diseases [9], [12], however the role of these pathways in PAH and in SSc-related vasculopathy has not yet been explored.

Endothelial cells constitute a first line of defense protecting tissues from injury. Elevated production of ET-1 is a common characteristic associated with endothelial cell dysfunction in various pathological conditions, including pulmonary arterial hypertension [33]. Previous studies have shown that HLA-B35 is associated with an increased risk for developing PAH in patients with scleroderma (SSc) [15]. The current study further supports the potential pathogenic role of HLA-B35 in upregulating ET-1 production and clarifies the molecular mechanism involved in this process in endothelial cells. In addition, this study raises an intriguing possibility that chronic activation of the eIF2α/ATF4 pathway could contribute to the disease pathogenesis. Although, we were able to demonstrate, activation of ATF4 in selected skin biopsies of patients with lcSSc, absence of full clinical data, including levels of circulating ET-1 and presence of HLA-B35 antigen, precluded proper analyses of these samples. This limitation may be addressed in future studies with a larger set of fully characterized samples from patients with lcSSc.

## Supporting Information

Figure S1 **Treatment with mouse monoclonal anti-MHC class I blocking antibody did not affect ET-1 and ATF4 mRNA levels in HDMECs transfected with HLA-B35.** PPET-1 (right panel) and ATF4 (left panel) mRNA after HLA-B35 (or HLA-B8) treatments with increasing dose of mouse monoclonal anti-MHC class I blocking antibody (W6/32) in HDMECs. Confluent dishes of HDMECs were transduced with 10 MOI of Adenovirus encoding HLA-B35/GFP (Ad-HLA-B8/GFP) for 24 h and then with increasing dose of W6/32 (0.1–10 µg/ml) for the following 24 hours. Total RNA was extracted and mRNA levels of PPET-1 and ATF4 were quantified by quantitative RT-PCR. Expression of the housekeeping gene β-actin served as an internal positive control in each assay performed. After measurement of the relative fluorescence intensity for each sample, the amount of each mRNA transcript was expressed as a threshold cycle value.
(TIF)
